# Peroxisome Proliferator-Activated Receptor Delta: A Conserved Director of Lipid Homeostasis through Regulation of the Oxidative Capacity of Muscle

**DOI:** 10.1155/2008/172676

**Published:** 2008-09-22

**Authors:** Pieter de Lange, Assunta Lombardi, Elena Silvestri, Fernando Goglia, Antonia Lanni, Maria Moreno

**Affiliations:** ^1^Dipartimento di Scienze della Vita, Seconda Università degli Studi di Napoli, Via Vivaldi 43, 81100 Caserta, Italy; ^2^Dipartimento delle Scienze Biologiche, Sez. Fisiologia ed Igiene, Università degli Studi di Napoli “Federico II”, Via Mezzocannone 8, 80134 Napoli, Italy; ^3^Dipartimento di Scienze Biologiche ed Ambientali, Università degli Studi del Sannio, Via Port'Arsa 11, 82100 Benevento, Italy

## Abstract

The peroxisome proliferator-activated receptors (PPARs), which are ligand-inducible transcription factors expressed in a variety of tissues, have been shown to perform key roles in lipid homeostasis. In physiological situations such as fasting and physical exercise, one PPAR subtype, PPARδ, triggers a transcriptional program in skeletal muscle leading to a switch in fuel usage from glucose/fatty acids to solely fatty acids, thereby drastically increasing its oxidative capacity. The metabolic action of PPARδ has also been verified in humans. In addition, it has become clear that the action of PPARδ is not restricted to skeletal muscle. Indeed, PPARδ has been shown to play a crucial role in whole-body lipid homeostasis as well as in insulin sensitivity, and it is active not only in skeletal muscle (as an activator of fat burning) but also in the liver (where it can activate glycolysis/lipogenesis, with the produced fat being oxidized in muscle) and in the adipose tissue (by incrementing lipolysis). The main aim of this review is to highlight the central role for activated PPARδ in the reversal of any tendency toward the development of insulin resistance.

## 1. INTRODUCTION

The modern Western lifestyle is characterized by excessive food intake and lack of physical exercise. This has led to obesity caused by a disturbance of lipid homeostasis, becoming one of the most prevalent and serious global chronic disorders. In lean organisms, fatty acids derived either from food or from hepatic lipogenesis are utilized as energy substrates by the heart and skeletal muscles. A strict physiological equilibrium between lipid availability and lipid consumption needs to be maintained to prevent development of both an impairment of insulin responsiveness and a metabolic dysfunction. In adult obesity and obesity-associated metabolic disorders (which have strict associations with type 2 diabetes, hypertension, and hyperlipidemia, and are often referred to as metabolic syndrome [1]), a disturbance of lipid homeostasis causes excess fat accumulation in various tissues (predominantly in adipose tissues, but also in other insulin-responsive organs, such as skeletal muscle and liver).

Skeletal muscle is quantitatively the largest organ in the body, and it contributes 30–40% of the resting metabolic rate in adults. It is a major site for the oxidation of fatty acids and glucose (accounting for approximately 80% of insulin-stimulated glucose uptake), and it exhibits a remarkable flexibility in its usage of fuel. One notable aspect of skeletal muscle plasticity is the specificity of its structural, biochemical, and functional adaptations to a given stimulus [2]. In view of the above features, it is perhaps not surprising that the predominant feature of type 2 diabetes is insulin resistance in skeletal muscle [3, 4].

The peroxisome proliferator-activated receptors (PPARs), which are ligand-inducible transcription factors expressed in a variety of tissues, have been shown to perform key roles in lipid homeostasis. In physiological situations such as fasting [5] and physical exercise [6], one PPAR subtype, PPAR*δ*, triggers a transcriptional program in skeletal muscle leading to a switch in fuel usage from glucose/fatty acids to solely fatty acids, and thereby drastically increasing this tissue's oxidative capacity. In addition, recent evidence has highlighted the possibility that activating PPAR*δ* in human subjects could increase skeletal muscle's oxidative capacity and so reverse metabolic abnormalities [7]. In mouse models, PPAR*δ* has been shown to play a crucial role in whole-body lipid homeostasis as well as in insulin sensitivity, and to be predominantly active in skeletal muscle (as an activator of fat burning [8, 9]) but also in the liver (where it can activate glycolysis/lipogenesis, with the produced fat being oxidized in muscle [10]) and in the adipose tissue (by incrementing lipolysis [11]). Thus PPAR*δ* activation provides a multiorgan “energy substrate-switching” phenotype that triggers tissue-specific transcriptional programs, and in which skeletal muscle plays a crucial role by reducing fat content.

From the current data presented in the literature, a central role for activated PPAR*δ* can be deduced in skeletal muscle, liver, and white adipose tissue (increased fat oxidation in muscle, increased carbohydrate catabolism and fat synthesis in the liver, and increased lipolysis in white adipose tissue) in the reversal of any tendency toward the development of insulin resistance. Following a brief description of the structure, the mode of activation and the action of the PPARs, this review aims to highlight the multiorgan energy switching role of PPAR*δ* and its ultimate impact on insulin resistance. Figure 1 represents an overview of the central role played by PPAR*δ* in the use of fatty acids as fuel by enhancing: (a) their oxidation in skeletal muscle (described in Section 3), (b) their synthesis from glucose in the liver and their subsequent release (described in Section 4), and (c) their release from the white adipose tissue (described in Section 5).

## 2. PPARS, NUCLEAR RECEPTORS ACTIVATED BY FATTY ACIDS

PPARs are nuclear receptors that act as ligand-inducible transcription factors. The three known isoforms PPAR *α*, *β* (also termed *δ*) , and *γ* display tissue-specific expressions and possess different gene-regulatory profiles. PPAR*γ* is a key regulator of adipose development and adipose insulin sensitivity [12], whereas PPAR*α*-regulated genes are involved in hepatic lipid oxidation [13]. The PPAR*δ* isoform, the function of which has only recently been elucidated and will be discussed in detail in this review, is predominantly expressed in skeletal muscle (where it induces fatty acid oxidation), but it is also expressed in brain, heart, liver, adipose tissue, and small intestine [14, 15].

It is generally known that PPARs heterodimerize with the retinoid X-receptor (RXR) and bind to a specific DNA sequence, (a sequence termed peroxisome proliferators response element (PPRE), that is found in a variety of genes involved in lipid and carbohydrate metabolism, inflammation, and cell proliferation and differentiation) [16, 17]. However, alternative mechanisms exist. Recently, an interplay has been reported between PPAR*δ* and thyroid hormone receptor *β* (TR*β*) in the activation of the gene encoding uncoupling protein 3 (UCP3) [18] in rat skeletal muscle as well as in cotransfection experiments in rat L6 myoblasts containing a reporter construct driven by the rat UCP3 promoter. Activation of UCP3 gene transcription in vivo by thyroid hormone (T3) requires the presence of fatty acids, while in the absence of fatty acids this transcription can be restored by the PPAR*δ* agonist L165,041 [18]. The UCP3 gene promoter has been shown to contain a noncanonical thyroid hormone response element (TRE) termed TRE1 that is conserved from rodents to humans [18, 19], and this response element is also recognized by PPARs [19]. Interestingly, fatty acid responsiveness after T3 treatment was only observed in cells transfected with the rat UCP3 promoter, which suggests a species-specific regulation [18].

Dietary fatty acids and fatty acid derivatives are the natural ligands of PPARs, which display the greatest preference for monounsaturated and polyunsaturated fatty acids (MUFAs and PUFAs, resp.), as demonstrated by means of various ligand-binding assays [20, 21]. The fact that each PPAR activates a different gene program, despite their overlapping expressions, would seem to suggest ligand-specificity for each PPAR. Indeed, the structure of the ligand-binding pocket differs considerably among the various PPARs as revealed by X-ray crystal-structure analysis [21, 22]. Nevertheless, natural fatty acids can be ligands of all three PPAR isoforms. It is well known that binding of the ligand promotes a conformational change that is permissive for interactions with tissue-specific coactivator proteins, allowing nucleosome remodelling and activation of the transcription of cell type-specific target genes [21, 23]. It is, therefore, conceivable that a given fatty acid induces different conformational changes when binding to the ligand-binding pockets of the various PPAR subtypes. Given that the transcriptional activity induced by each PPAR subtype is cell type-specific [24], the different conformations induced following ligand binding may determine the cell-specificity of the different PPARs (through heterodimerization with different receptors and binding to cell-type specific cofactors). However, further research is needed to establish which natural ligands might activate each PPAR in a given cellular context.

## 3. ROLE OF PPAR*δ* IN SKELETAL MUSCLE: A SWITCH TO FAT OXIDATION

### 3.1. PPAR*δ*-induced fuel switching evidenced by its overexpression or ablation and by the use of synthetic ligands in rodents

In skeletal muscle, the relatively high expression of PPAR*δ* (at 10- and 50-fold higher levels than PPAR*α* and PPAR*γ*, resp.; [15, 25]) as well as its preferential expression in oxidative rather than glycolytic myofibers [9], has led to the suggestion that this receptor isoform may be involved in promoting the utilization of fatty acids as fuel. Indeed, treatment of rat L6 cells with the highly specific PPAR*δ* agonist GW0742 has been shown to increase fatty acid oxidation and induce expression of several lipid regulatory genes [26]. In addition, treatment of C2C12 cells with GW0742 [27] or with another the PPAR*δ*-specific agonist (GW1516 [28]) induced expressions of genes involved in lipid catabolism and energy uncoupling in skeletal muscle cells [29]. However, although an in vivo magnetic resonance spectroscopy (MRS) study of rats treated with the latter agonist revealed increased lipid metabolism, no change in mitochondrial energy coupling was detected efficiency despite an increased UCP3 expression [29]. Skeletal muscle has the capacity to adapt its structure to metabolic changes, as indicated by changes in the myosin type and a subsequent shift in the number and type of muscle fibers. An increased demand for fat metabolism is reflected by a shift in fiber-type away from the fast, glycolytic form (type II) toward the slow-oxidative form (type I) [2]. PPAR*δ* has emerged as an important stimulus in the induction of this fiber shift. Indeed, studies on transgenic mice harboring a constitutively activated form of PPAR*δ* (VP16-PPAR*δ*) have clearly shown an increase in skeletal muscle lipid metabolism as well as the formation of type I fibers [9]. Mice overexpressing peroxisome proliferator-activated receptor *γ* coactivator 1 *α* (PGC-1*α*), which activates PPAR*δ* via a direct protein-protein interaction [30], have been shown to possess a high content of type I fibers [31]. However, experiments on mice overexpressing VP16-PPAR*δ* have revealed that type I fiber formation can be directly stimulated by PPAR*δ* without an induction of PGC-1*α* [9]. Nevertheless, in physiological situations, an upregulation of PGC-1*α* is likely to be involved in the early events leading to muscle-fiber shifts, since PGC-1*α* is a coactivator of the PPARs. Indeed, PGC-1*α*-null mice show clear muscle dysfunction [32], and evidence that PPAR*δ* induces an expression of PGC-1*α* has come from treatment of mice with GW1516 [8] as well as from a study in which skeletal muscle C2C12 myocytes transfected with a PGC-1*α* promoter-driven reporter construct were treated with the same ligand [33]. A wild-type PPAR*δ* transgene (specifically overexpressed in mouse skeletal muscle, but not constitutively activated) has been shown to promote a net increase in the number of fibers with an oxidative metabolic capability through an increase in fiber numbers in soleus and tibialis anterior muscle, while in plantaris muscle the increase was more closely related to a shift from glycolytic to more oxidative fibers [34]. Interestingly, this nonactivated PPAR*δ* transgene failed to induce the formation of type I fibers in skeletal muscle [34]. In this case, despite its high expression, actual activation of the transgene would depend on the presence of natural ligands, such as fatty acids. As the fatty acid concentrations fluctuate, fatty regulation of PPAR*δ* transcription is likely to be highly regulated.

This raises the question as to whether, instead of overexpression, increasing the availability of ligand (natural or artificial) would induce fuel switching as well as fiber switching toward type I fibers. Indeed, a fuel-switching role of PPAR*δ* activation has been demonstrated by incubating rat isolated skeletal muscle strips with the agonist GW1516 for 24 hours [35]. This led to an increased use of fatty acids over glucose, as reflected by increased fatty acid oxidation and reductions in glucose oxidation, glycogen synthesis, lactate release, and glucose transport. Interestingly, this switch was independent of insulin stimulation or fiber type [35]. The PPAR*δ* agonist GW610742 also induced this fuel switch and in addition triggered a genetic program toward initiation of muscular atrophy without compromising mitochondrial activity in rat skeletal muscle [36]. Furthermore, a somatic gene transfer of PPAR*δ* into adult rat fibers has recently been shown to lead to activation of fuel switching as well as to a shift in the existing fiber profile toward the “slow,” oxidative phenotype, an effect that caused the number of type I fibers in the extensor digitorum longus (EDL) muscle to be tripled after 14 days [37]. From these experiments, it is clear that PPAR*δ* rapidly programs all fiber types in skeletal muscle to oxidize fatty acids.

### 3.2. Evidence supporting a role for activated PPAR*δ* in mediating fuel switching in human skeletal muscle: data from in vitro and clinical studies

Recent studies have revealed clear roles for PPAR*δ* in the regulation of lipid and glucose metabolism in human skeletal muscle [7, 38]. PPAR*δ* stimulates the expression of genes involved in (a) increasing of lipid oxidation (fatty acid binding protein 3 (FABP3) and CPT1) and (b) reducing carbohydrate oxidation (pyruvate dehydrogenase kinase 4 (PDK4)) in human skeletal muscle [38], as it does in rodents [5, 8–10]. These in vitro human skeletal muscle data with GW1516 support the long-known observation that an increase in fatty acid oxidation reduces the glucose utilization of isolated muscle reflecting the mutual inhibition in the metabolism of substrates involved in the glucose-fatty acid cycle [35, 36, 39]. Recent data from a clinical study indicate that this situation holds true in human subjects. A statistically significant reduction in fasting insulin levels was observed in a study performed on moderately obese men given a dose of 10 mg o.d. of GW1516 was given for 2 weeks [7]. These subjects also showed decrease fasting plasma nonesterified fatty acid (NEFA) concentrations and increased expression of CPT1b in muscle. Interestingly, GW1516 treatment slightly reduced the expression of PPAR*δ*, showing that overexpression of the receptor itself is not necessary for the induction of PPAR*δ*-mediated effects, the resident levels of the receptor protein being sufficient. In contrast, similar treatment with a PPAR*α* agonist (GW590735) did not result in any change in plasma insulin levels, nor did it cause a significant increase in CPT1b mRNA [7].

### 3.3. PPAR*δ*, a regulator of fuel use in skeletal muscle under physiological conditions

Since fasting promotes increased utilization of fatty acids, fasting might also regulate PPAR*δ* expression. However, the initial reports appearing in the literature did not seem to confirm this. For instance, a 24-hour fasting period was found not to upregulate PPAR*δ* in rat skeletal muscle [40], and our group even reported reduced levels of PPAR*δ* (and PPAR*α*) in gastrocnemius muscle from 48-hour-fasted rats [25]. Decreased expressions of PPAR*δ* and PPAR*α* upon 48 hours of fasting have recently been reported in humans, too [41]. In contrast, in mice, skeletal muscle PPAR*δ* levels were found to be upregulated after a 24-hour fast [42]. One explanation is that studying the responses to physiological stimuli by making single time point measurements may give misleading results, due to possible transient modifications. Indeed, time course studies have shown that PPAR*δ* actually is upregulated in fasted rat skeletal muscle, but within the first 6 hours [43]. This upregulation of PPAR*δ* (and of PGC-1*α*) during fasting is, however, transient [43], downregulation (after the initial upregulation at 6 hours to around or below the control levels being evident at 48 hours). Data showing that rapid nuclear accumulations of both PGC-1*α* and PPAR*δ* upon food deprivation [43], and their physical interaction within the nucleus [30], occur concomitantly with increases in fatty acid levels and an increase in the expression of myosin heavy chain Ib (MHC Ib), underline the role of PPAR*δ* as a key regulator of fatty acid metabolism and muscle fiber switching (in concert with its coactivator, PGC-1*α*).

Following the nuclear accumulation of PPAR*δ*, its target genes (such as carnitine palmitoyl transferase 1b (CPT1b), mitochondrial thioesterase I (MTE I), and UCP3) are upregulated simultaneously, and so is the rate of mitochondrial fatty acid oxidation [43]. In starved mice, the mRNA for a member of the FOXO family, FKHR (forkhead homolog in rhabdomyosarcoma), is upregulated rapidly and transiently (starting within 6 hours, peaking at 12 hours, and decreasing at 24 hours), and this is followed by an upregulation of FKHR protein and a nuclear accumulation of nonphosphorylated FKHR levels with a consequent upregulation of its target gene pyruvate dehydrogenase kinase 4 (PDK4) [44]. In mouse skeletal muscle, PDK4 has been shown to be a target of PPAR*δ*, since it is activated in vivo by GW1516 [8]. This kinase plays an important role in the switching from glucose usage to fat usage since it phosphorylates the E1 component of the pyruvate dehydrogenase (PDH) complex, thereby downregulating carbohydrate (CH) oxidation [45]. Similarly, in human skeletal muscle, PDK4 mRNA and protein levels have been found to be elevated at both 24 hours and 48 hours of fasting, whereas at these time points the FOXO1 mRNA/protein levels were unchanged [41]. However, it is possible that regulation of the mRNA/protein levels of FOXO1 (a target of PGC-1*α* [46], which are transiently regulated during fasting in rats [40]) is a transient event preceding upregulation of PDK4 mRNA and protein in humans, too. If so, such transient regulatory changes may have been missed by measuring only at 24 hours and 48 hours of starvation in humans. At the 48-hour time point of starvation, PPAR*δ* mRNA levels in the human vastus lateralis muscle were decreased [41], a finding in line with the decreased levels of PPAR*δ* mRNA [25] and nuclear protein [43] at this time point in fasting rat gastrocnemius muscle. In the rat, this decline was preceded by a rapid rise in the mRNA and protein levels of this transcription factor, elevated levels being detected at 6 hours and 12 hours of food deprivation [43]. Unfortunately, these time points were not investigated in the human study [41]. Thus kinetic studies in the fasting situation, in rodents as well as in humans, have made it clear that the expression of PPAR*δ*, and that of its target genes, is tightly regulated. These results offer an explanation for the rapid structural and metabolic changes favoring an increased use of lipids as fuel that occur in this condition.

The reported kinetics of the PPAR*δ* upregulation occurring during the recovery period after exercise-imposed energy stress in humans are in line with those seen in the fasting rat; a single exhaustive bout of cycling increasing PPAR*δ* mRNA and protein expression within 3 hours after completion of the exercise [47, 48]. Regular physical training, which elevates the levels of PPAR*δ* and PGC-1*α*, leads to increases in both mitochondrial capacity and insulin sensitivity [34, 49–51], effects similar to those seen after PPAR*δ* activation. The observations made in exercise and fasting experiments showing that PPAR*δ*-expression kinetics are rapid, and the changes almost immediate, are supported by PPAR*δ* acutely bringing about the fuel switching effects inpre-existing adult rat muscle fibers (as demonstrated by short-term agonist treatment [35, 36] and somatic PPAR*δ* gene transfer [36]). Recently, a direct role for PPAR*δ* in the suppression of glucose oxidation in fasting skeletal muscle has been shown by Nahlé et al. [52]. First, the authors demonstrated that deficiency of the fatty acid translocase CD36 (mediating muscle fatty acid uptake during fasting, [5]) blunts fasting induction of FOXO1 and PDK4 and the associated suppression of glucose oxidation in mouse skeletal muscle [52]. Next, they demonstrated that loss of PPAR*δ* abolishes the fasting induction of muscle FOXO1 and PDK4 in vivo [52]. As the authors identified several PPRE sites in the FOXO1 promoter, these results suggest that CD36-dependent activation of PPAR*δ* results in the trascriptional regulation of FOXO1 as well as PDK4 in fasted mice.

Taken together, the control of fuel use by activated PPAR*δ* has emerged to be crucial for the rapid metabolic adaptation of skeletal muscle to energy stress.

## 4. ANTIGLYCEMIC ACTION OF PPAR*δ* IN LIVER: CONVERTING GLUCOSE INTO FAT

At first glance, the above described PPAR*δ*-mediated fuel switching in skeletal muscle would be expected to give rise to insulin resistance, since a preferential uptake and oxidation of fatty acids (FFAs) over glucose (mediated by PPAR*δ* stimulation in skeletal muscle) would lead to an accumulation of blood glucose, muscle being a major player in blood-glucose homeostasis [1, 2]. However, as well as stimulating skeletal muscle fatty acid oxidation, PPAR*δ* plays a surprising role in ameliorating hyperglycemia. It does this by increasing hepatic glucose flux through the pentose phosphate pathway and by enhancing fatty acid synthesis, the fatty acids being destined for oxidization in muscle [10]. Whereas PPAR*δ*-deprived mice are metabolically less active and glucose intolerant, db/db mice treated with GW1516 show increased levels of CPT in muscle [10] (similar effects of this agonist being reported in [8, 9]). This effect on CPT is indicative of increased fatty acid oxidation, so it was a surprising finding that gene array analysis revealed increased expression of gene clusters involved in fatty acid synthesis and the pentose phosphate cycle in the liver [7], both pathways using glucose or its metabolites as substrates. The authors [10] suggested that PPAR*δ* may increase glucose catabolism through these processes, with the result that peripheral insulin sensitivity may be improved [10]. Indeed, GW1516-treated db/db mice showed an improved performance in the glucose tolerance test, and also showed a tendency toward lowered fasting serum insulin levels [10].

## 5. ROLE FOR PPAR*δ* IN WHITE ADIPOSE TISSUE: INCREASING LIPOLYSIS

Interestingly, adipocyte hypertrophy induced by high-fat diet was accompanied by increased cannabinoid receptor type 1 (CB1R) expression and by a decrease in PPAR*δ* expression in adipose tissue [11]. Exercise attenuates adipocyte hypertrophy and normalizes expression of CB1R and PPAR*δ*. Functional cross-talk between CB1R and PPAR*δ* is established by RNA interference experiments in 3T3-L1 preadipocytes. For example, selective silencing of PPAR*δ* by RNA interference significantly increased CB1R and increased adipocyte differentiation and adenovirus-mediated overexpression of PPAR*δ* reduced CB1R expression [11]. The role of CB1R in obesity is well established [53]. Depletion of CB1R in knockout mice is known (in animals fed a high-fat diet) to reduce obesity through increased lipolysis [53].

The simultaneous regulation of skeletal muscle fatty acid oxidation and adipose proliferation by PPAR*δ* underlines the powerful role this receptor may play in preventing weight gain in physiological situations.

## 6. CONCLUSIONS

Recent evidence shows that the fuel-switching role of PPAR*δ* in skeletal muscle is conserved from rodents to humans. This receptor is crucial for a modulation of skeletal muscle flexibility that directs this tissue toward the use of fatty acids as fuel, an effect with rapid kinetics. It is becoming increasingly clear that even though the fat oxidation-inducing effect of PPAR*δ* is exerted in skeletal muscle, this receptor also activates transcriptional programs in other tissues (such as adipose tissue, in which PPAR*δ* directly inhibits proliferation and induces lipolysis), thereby channelling the fat consumed in the diet directly to muscle for oxidation. In addition, in an action that serves to prevent insulin resistance developing as a consequence of a reduction of carbohydrate oxidation in muscle, the liver is activated to form fat from glucose, thereby both allowing skeletal muscle to oxidize more fat and concomitantly lowering blood glucose levels. PPAR*δ* is emerging as a crucial nuclear receptor for the multiorgan regulation of whole body fuel turnover, with skeletal muscle as the central organ in the burning of fat and the consequent prevention or reduction of obesity (see Figure 1). These features make PPAR*δ* a good candidate as a central target for the future treatment of metabolic disturbances linked to obesity and insulin resistance.

## Figures and Tables

**Figure 1:** Central, fuel-switching mechanisms by which PPAR*δ* increases the use of fatty acids in skeletal muscle without provoking insulin resistance. Dotted arrow: indirect effect. For abbreviations, the reader is referred to the text.
